# Impacts of Daily Life and Job Satisfaction on Social Participation of Persons with Visual Impairment

**DOI:** 10.1155/2023/6475756

**Published:** 2023-07-22

**Authors:** Hyeong-min Kim, Sung-min Son

**Affiliations:** ^1^Department of Occupational Therapy, Gimcheon University, Gimcheon, Republic of Korea; ^2^BK21 FOUR R&E Center for Learning Health Systems, Korea University, Seoul, Republic of Korea

## Abstract

**Objective:**

This study is aimed at providing baseline data for improving the social participation of persons with visual impairment by verifying the impacts of daily life satisfaction and job satisfaction on their social participation.

**Methods:**

This study utilized data from the 5th survey of the 2nd wave of the Panel Survey of Employment for the Disabled (PSED) provided by the Korea Employment Agency for Persons with Disabilities (KEAD). Of the 511 persons with visual impairment who participated in the panel survey, 151 people who met the inclusion criteria were selected as the research subjects. This study compared social participation, job satisfaction, and daily life satisfaction, which were validated by experts' review, consulting, and research at the KEAD.

**Results:**

Daily life satisfaction and job satisfaction of persons with visual impairment had positive correlations with social participation. Job satisfaction had a statistically significant impact on social participation. Additionally, the stability of employment and monthly income were the variables affecting social participation.

**Conclusion:**

The result drawn in this study can be applied as basic data related to the social participation of people with visual impairment.

## 1. Introduction

Disability has a major impact on daily life and participation in the activities of daily life, such as motor function, defecation, urination, bathing, and moving [1]. Recently, the disability paradigm has gradually emphasized environmental factors and, changes have resulted, such as deinstitutionalization, the spread of independent living for persons with disabilities, and an increase in the desire for social participation [2]. However, negative perceptions and attitudes toward persons with disabilities remain because of low expectations for their achievements and the tendency that they perceive themselves to be potentially rejected by society, which reduces their social participation [3–5].

Social participation indicates participation in the interweaving of occupations to support desired engagement in community and family activities as well as those involving peers and friends that support social interdependence [6]. Recently, there has been increasing recognition of participation as a fundamental concept in the field of occupational therapy, understanding its heightened importance for health [7, 8]. Occupational therapy helps clients who have difficulties in social participation due to physical and environmental factors, etc., to improve their lives through occupation and to participate in local communities [9].

Variables that can quantify social participation and local community integration include life satisfaction and job satisfaction [10]. Pursuing satisfaction in daily life is the basic goal of all human beings, and living a high-quality life may be the greatest concern of humans [11]. For satisfaction with daily life, it is important for persons with disabilities to actively participate in social activities in community life [2]. Additionally, the pleasure brought by work-oriented social activities and daily life satisfaction related to them has very important meanings for their welfare [12].

Productive activities such as employment are important for self-realization, giving meaning to their lives, and local community integration, in addition to a means that increases income [13]. Acknowledging the significance of job satisfaction for both health and productivity [14], it is imperative to incorporate this aspect into the practice and policy framework concerning persons with disabilities [15]. This recognition is closely intertwined with their overall quality of life. Job satisfaction is defined as an emotional state related to reaching one's goals. It promotes self-confidence and supports the development of one's identity [16]. Job satisfaction is an important factor in inducing organizational commitment [17]. Moreover, it has value as an important variable that mediates social participation in an individual's daily life by acting as an implicit and explicit motivating factor in inducing social participation [18]. Concerning the perception of the job, the attitudes and values of persons with visual impairment can be important factors to form job satisfaction, which can directly affect successful social participation.

Social participation and productive activity are important in people's lives, but most persons with disabilities have difficulty interacting with and participating in the local community [19]. Among disabilities, visual impairment significantly impacts the body and daily functions [20, 21], and often, those with visual impairment have difficulty leading an independent life due to various restrictions in daily life activities [22]. Furthermore, individuals with vision loss experience a diminished capacity to engage in functional activities [23, 24], consequently impacting their participation across various domains of occupation, including leisure and social activities [25].

Previous studies examining social participation among people with visual impairment have explored various approaches, such as the implementation of a multidisciplinary group rehabilitation program [26] and the promotion of lifestyle habits [27], the quality of life [28], the correlation of social participation of the elderly [29], the experience of discrimination in daily life [30], the determinants of social participation [22], occupational therapy intervention to improve social participation [25], and the relationship between double sensory loss and social participation [31]. In recent times, there have been growing calls for support and measures that take into account the overall job satisfaction and subjective experiences of persons with disabilities in their daily lives [10]. However, there remains a scarcity of published evidence that specifically addresses the daily life and job satisfaction of persons with visual impairment and their impact on social participation. This research gap underscores the need for new insights and empirical findings in this area. By addressing this gap, the present study is aimed at contributing to the existing knowledge base and providing valuable insights into the relationship between daily life satisfaction, job satisfaction, and social participation among people with visual impairment.

Recognizing the importance of understanding the relationship between vision impairment and social participation, this study is aimed at contributing to the development of future interventions that promote social engagement and enhance the overall health and well-being of people with visual impairment [32]. By comprehensively exploring variables that facilitate functional independence, integration into local communities, and improvements in quality of life, the study seeks to adopt an integrated approach [12]. The primary objective of this study is to identify potential alternative approaches, beyond traditional mediation strategies, and to facilitate active social participation among persons with visual impairment. Specifically, the study is aimed at demonstrating the impacts of daily life satisfaction and job satisfaction on the social participation of persons with visual impairment. By highlighting these influences, the research endeavors shed light on possible avenues for enhancing social engagement and promoting the active involvement of people with visual impairment in society.

## 2. Methods

### 2.1. Participants

This study utilized data from the 5th survey of the 2nd wave of the PSED (Panel Survey of Employment for the Disabled) conducted by the Korea Employment Agency for Persons with Disabilities (KEAD). The inclusion criteria for selecting the research sample were as follows:

(1) people with visual impairment, (2) samples who responded to the survey by themselves, (3) samples that did not have any unanswered questions or responses marked as “I don't know” for the variables measured in this study, (4) samples aged between 19 and 65 years. Out of the 511 persons with visual impairment who participated in the PSED, 151 individuals met the abovementioned sampling conditions and were selected as the final research subjects for this study.

### 2.2. Analysis Material and Survey Method

The primary data source utilized in this study is the PSED (Panel Survey of Employment for the Disabled), conducted annually by the Employment Development Institute of the Korea Employment Agency for persons with disabilities. The PSED is a longitudinal survey aimed at collecting data on the economic activity of persons with disabilities. Its purpose is to provide baseline data for the development and evaluation of employment policies for persons with disabilities while investigating various individual and environmental factors that influence their employment outcomes [33].

The PSED database comprises 11 surveys, covering a range of topics related to employment and disability. These surveys include basic panel information, economic activity status determination, wage workers/nonwage workers/unemployed classification, efforts and support for employment, occupational ability, employment attitude and environment, daily life and quality of life, and general household matters. Each of the 11 areas is further divided into detailed investigation contents. Out of the 11 domains covered in the survey conducted by the PSED, the present study focused on specific variables related to job satisfaction among wage workers. The analysis primarily utilized data on social participation and daily life satisfaction from the domains of daily life and quality of life. These variables were selected as key factors for examining the relationship between job satisfaction and overall well-being and satisfaction in daily life among the study participants.

This study primarily utilized Tablet PC-Assisted Personal Interviewing (TAPI) conducted on a tablet PC. The TAPI program was designed with preestablished logic to minimize errors and inaccuracies that could arise from complex questionnaire items. This design allowed the investigator to promptly identify incorrect responses. Prior to the interviews, the investigator consulted with the participants to arrange a suitable visiting schedule. Face-to-face interviews were then conducted, and the responses were entered directly into the tablet PC. However, in cases where face-to-face interviews were declined due to the COVID-19 pandemic, online and telephone surveys were conducted as alternatives. During telephone surveys, the surveyor entered responses directly into a tablet PC, and if the survey was interrupted due to a prolonged call, it was resumed later at a convenient time for the participant. The online survey used the same set of questions as the face-to-face interviews. Participants were provided with individual URLs to participate in the online survey, and the investigator was available to address any immediate inquiries or concerns from the participants.

### 2.3. Social Participation

Social participation encompasses engagement in both formal and informal social groups, gatherings, and ceremonies. This can include activities such as attending religious events, graduation ceremonies, weddings, and other social gatherings where individuals interact and actively participate in social contexts, which consists of a single question, “To what extent do you think you participate in these ceremonies and activities?”. The question consisted of a 4-point Likert scale with “I never participate=1 point,” “I tend not to participate=2 points,” “I tend to participate=3 points,” and “I participate often=4.” The total score for each question serves as an indicator of the level of social participation, with a higher score reflecting a better degree of social participation. Cronbach's *α* was .742 in this study.

### 2.4. Job Satisfaction

The question was developed by adapting and condensing the Minnesota Satisfaction Questionnaire (MSQ) from the Vocational Psychology Research Institute at the University of Minnesota as well as the Job Description Index created by Smith et al. [31–34]. By utilizing these established measures, the study is aimed at assessing participants' levels of job satisfaction accurately. This job satisfaction measure consisted of 10 questions in total, including (1) wages and income, (2) employment stability, (3) details of work, (4) working environment, (5) working hours, (6) individual's development potential, (7) communication and interpersonal relationships, (8) fairness in personnel appraisal, (9) welfare, and (10) consideration and convenience for the disabled. Each question in the survey was rated on a 5-point Likert scale, ranging from “very low” assigned 1 point to “very high” assigned 5 points. A higher total score for each question indicates a higher level of job satisfaction. Cronbach's *α* of this study was .874.

### 2.5. Daily Life Satisfaction

For daily life satisfaction, eight questions on daily life satisfaction were used: (1) relationships with family, (2) relationships with friends, (3) living place, (4) health conditions these days, (5) monthly income (pocket money), (6) leisure activities, (7) work being done, and (8) satisfaction with marital life. Each question in the survey was rated on a 5-point Likert scale, where “very unsatisfied” was assigned 1 point and “very satisfied” was assigned 5 points. A higher total score for each question indicates a higher level of daily life satisfaction. In this study, Cronbach's *α* was .856.

### 2.6. Control Variable

Based on the preceding studies of the social participation of persons with disabilities, sex, age, educational level, the severity of the disability, and the existence of a spouse were set as control variables [32, 33, 35, 36]. Sex (woman = 0, man = 0), disability severity (minor = 0, major = 1), and the existence of a spouse (yes = 0, no = 1) were processed as dummy variables. In the dummy variables, the reference group was “man” by sex; “minor” by disability severity; and “yes” by the existence of a spouse. For age (15-29 = 1, 30-39 = 2, 40-49 = 3, 50-59 = 4, 60-68 = 5) and educational level (less than middle school graduation = 1, under high school graduation = 2, more than university graduation = 3), continuous variables provided by the PSED were used.

### 2.7. Statistical Analysis

The data were analyzed using SPSS WIN 22.0. Descriptive statistics were utilized to analyze the general characteristics of the study subjects. Pearson's correlation coefficient was employed to examine the relationships between the general characteristics of visually impaired individuals, job satisfaction, daily life satisfaction, and social participation. Lastly, a multiple linear regression analysis was conducted to investigate the impact of each variable on social participation. Statistical significance was determined at alpha = .05.

## 3. Results

### 3.1. Research Subjects' General Characteristics

The demographic and sociological characteristics of the respondents of this study were investigated, and the results are as follows. There were more men than women in the visually impaired samples, and most were 50-59 years old. Most were high school graduates or higher, and most had minor disabilities (Table 1).

### 3.2. Correlation among the Variables That Affect Social Participation

In this study, Pearson's correlation analysis was conducted to examine the relationships among the variables that influence social participation. The purpose of this analysis was to assess the extent of correlation between these variables and gain insights into their interrelationships. As a result of the analysis, daily life satisfaction (*r* = .297, *p* < .001) and job satisfaction (*r* = .310, *p* < .01) had a positive correlation with social participation (Table 2).

### 3.3. Causal Relationships of the Subfactors of Daily Life Satisfaction with Social Participation

To examine the relationship between the subfactors of daily life satisfaction of persons with visual impairment and their social participation, a multiple linear regression analysis was performed (as presented in Table 3). The aim of this analysis was to determine the extent to which the subfactors of daily life satisfaction predict social participation among people with visual impairment. In all variables, the tolerance was higher than the VIF value, which was lower than 10.0, so there was no problem with multicollinearity. Based on the Durbin-Watson test, the obtained *d* value of 1.985 indicates the absence of autocorrelation in the data. This means that the residuals in the regression analysis are independent and do not display any systematic pattern of correlation. Consequently, the regression analysis results can be deemed reliable and suitable for further interpretation. As a result of analyzing the impact of daily life satisfaction of persons with visual impairment on social participation, the *F* value was 10.840 (*p* < .001), which showed that this regression model was appropriate, and the adjusted value of the coefficient of determination was adj. = .362. Of them, monthly income (*B* = .195, *p* < .01) had a statistically significant impact on the social participation of people with visual impairment (Table 3).

### 3.4. Causal Relationship of the Subfactors of Job Satisfaction with Social Participation

To examine the relationship between the subfactors of job satisfaction of persons with visual impairment and their social participation, a multiple linear regression analysis was performed (as shown in Table 4). This analysis aimed to determine the extent to which the subfactors of job satisfaction predict social participation among persons with visual impairment. In all variables, the tolerance was higher than the VIF value, which was lower than 10.0, so there was no problem with multicollinearity. Based on the Durbin-Watson test, the obtained *d* value of 1.810 indicates the absence of autocorrelation in the data. This implies that the residuals in the regression analysis are independent and do not exhibit any systematic pattern of correlation. Therefore, the regression analysis results can be considered reliable and valid for further interpretation. As a result of an analysis of the impact of job satisfaction for people with visual impairment on social participation, the *F* value was 11.367 (*p* < .001), which showed that this regression model was appropriate, and the adjusted value of the coefficient of determination was adj. = .387. Of them, stability of employment (*β* = .252, *p* < .01) had a statistically significant impact on the social participation of persons with visual impairment (Table 4).

### 3.5. Causal Relationship among Variables Affecting Social Participation

The result of the regression analysis of the impacts of daily life satisfaction and job satisfaction of persons with visual impairment on social participation is like Table 5. To assess the presence of multicollinearity between the independent variables, tolerance and variance inflation factor (VIF) were analyzed. The results indicated that the tolerance values were greater than 0.10, and the VIF values were smaller than 10, indicating no multicollinearity among the independent variables. Additionally, the Durbin-Watson test was conducted to test the independence of the residuals. The obtained value of 1.653 suggested no autocorrelation in the data. These findings assure the validity of the regression analysis and provide confidence in the independence and reliability of the study results. As a result of an analysis of the influence on social participation, the *F* value was 11.519 (*p* < .001), which showed that this regression model was appropriate, and the adjusted value of the coefficient of determination was adj. = .388. Among the examined factors, the study ultimately revealed a statistically significant impact of job satisfaction (*β* = .159, *p* < .01) on the social participation of people with visual impairment (as shown in Table 5). This finding suggests that higher levels of job satisfaction are associated with increased social participation among persons with visual impairment.

## 4. Discussion

Social participation is significant for persons with disabilities, so it is considered the criterion for identifying successful rehabilitation [37]. Participating in meaningful social activities holds significant importance for the daily functioning and psychological well-being of individuals with vision loss. These activities contribute to their overall well-being and help them maintain a sense of purpose, connection, and fulfillment despite their visual impairment [25]. By engaging in meaningful social interactions and activities, people with visual impairment enhance their quality of life and experience greater satisfaction in their daily lives. In occupational therapy, participation has always been the main concern, and an occupational therapist is in a unique position that can contribute to the development and implementation of participation for both persons with disabilities and those without disabilities [38]. Thus, it is important to maintain or enhance the level of social participation of persons with visual impairment [22], and an occupational therapist should investigate and reveal the related variables to achieve this goal. This study was conducted to identify variables that affect the social participation of persons with visual impairment.

Building upon the theoretical contributing factors identified in Whetten's study [39], our research findings provide a theoretical contribution by proposing a novel relationship between daily life satisfaction, job satisfaction, and social participation among people with visual impairment. This new perspective enhances our understanding of the complex dynamics that influence the social participation of persons with visual impairment and contributes to the existing body of literature in this field. Therefore, the theoretical contribution is interesting for our readers.

The utilization of the PSED data in this study provides valuable insights into the process of entry of persons with disabilities into the labor market, their mobility within it, the characteristics of economic activity throughout their life cycles, and the changes in employment patterns and preferences. These data offer a comprehensive understanding of various factors that are pertinent to the development and evaluation of employment policies for persons with disabilities [30–33]. By leveraging the PSED data, researchers and policymakers can gain a holistic perspective on the establishment and assessment of employment policies aimed at promoting the inclusion and success of persons with disabilities in the workforce. This study is aimed at analyzing the effects of daily life satisfaction and job satisfaction on the social participation of people with visual impairment, and as a result, job satisfaction had a statistically significant impact on the social participation of persons with visual impairment. Since *B* has a positive sign, the higher job satisfaction, the more social participation becomes. Attempts have been made to compare and examine this research result; however, there have been few studies to understand the relationship between social participation and job satisfaction of persons with disabilities. There is a slight difference between the subjects and variables of the studies to compare; however, Yoo [40] reports that the higher the job satisfaction, the better the social relationship becomes, which partly supports the results of this study.

This study examines job satisfaction, concerning the social participation of persons with visual impairment. In the vocational rehabilitation area, the roles of occupational therapists include career counseling and evaluation, job competency improvement, job preparation and adaptation training, education and research, and subjective satisfaction improvement for the successful vocational life and social adjustment of persons with disabilities [41]. Therefore, the role of occupational therapists is crucial in the field of vocational rehabilitation to enhance their social adjustment and social participation. Occupational therapists play a significant role in supporting them in developing the necessary skills, providing interventions, and facilitating their successful integration into the workforce, ultimately promoting their overall social adjustment and participation. Occupational therapists should address the subjective job satisfaction perceived by persons with disabilities to induce successful social participation.

This study analyzed the impacts on social participation, with daily life satisfaction items as independent variables and monthly income (*β* = .195, *p* < .01) having a statistically significant impact on the social participation of persons with visual impairment. Previous studies supported these findings [42, 43] examining the factors influencing social participation among people with disabilities have consistently reported that higher monthly income is associated with increased levels of social participation. These findings align with the results of the current study, further supporting the notion that a higher monthly income positively influences social participation among persons with disabilities.

Employment stability (*β* = .252, *p* < .01) had a significant impact on the social participation of people with visual impairment. The ultimate purpose of welfare for persons with disabilities is employment, which can be evaluated by employment performance, and what is important along with employment is to maintain a job in terms of employment stability [44]. Furthermore, enhancing job satisfaction by ensuring employment stability and a steady income is crucial for promoting social participation and improving the quality of life for people with disabilities. The stability of employment and consistent monthly income are closely linked to the overall quality of life for persons with visual impairment and serve as important factors influencing their level of social participation. So occupational therapists should include these intervention targets in the process of vocational rehabilitation.

Alderfer's Existence-Relatedness-Growth Theory can also explain the results of this study. Schneider and Alderfer [45] argued that human needs are divided into existence needs, relatedness needs, and growth needs. The main variables affecting social participation identified by this study were monthly income and the stability of employment, which are consistent with existence needs, in other words, human beings' basic needs for survival, such as food, clothing, and shelter and occupational stability and economic security supporting them. Lee's study [46] of older adults reported that participation in economic activity contributes to increased life satisfaction, which was consistent with our study results. The study conducted by Yeum et al. [47] on disabled workers also found that job satisfaction acts as a mediating factor in the association between social networks and life satisfaction. These findings are consistent with the results obtained in our study, further supporting the relationship between job satisfaction, social network, and overall life satisfaction.

In occupational therapy, concern with functional ability and purposeful activity are unique features that allow the profession an important place in vocational rehabilitation practice [42]. Employment for persons with disabilities is a source of income, which is important for social participation [48]. Of the various experts in the vocational rehabilitation field, an occupational therapist can play a role in helping them secure stable employment and maintain a job, drawing on their potential as well as occupational characteristics according to the type of disability [49]. Furthermore, vocational rehabilitation helps persons with disabilities continue to play social roles and confirm their worth, allowing them to get a job [50]. Subjective job satisfaction, stability of employment, and monthly income are important in the lives of people with visual impairment as occupational beings. This study has significance in that it empirically verified that managing these variables well may be a measure for facilitating social participation for persons with visual impairment.

Despite the significance of this study, there are several limitations that should be acknowledged. Firstly, the use of secondary data in this study limited the ability to measure each variable precisely and generalize the findings. Future research should consider collecting data using standardized scales that specifically reflect the characteristics of the diseases in order to evaluate the relationship with participation in social activities more accurately. Secondly, the reliability of the variable of social participation was challenging to establish with a single question item. In this study, panel survey data based on longitudinal analysis was utilized, with a panel retention rate of 86.3% for the Panel Study of Entrepreneurial Dynamics (PSED). To address this, reliability was assessed by cross-validating data from the 3rd, 4th, and 5th waves of the PSED analyzing the time difference between panel survey responses. In future studies, it is important to design research that takes into account the limitations identified in this study. These limitations highlight the need for further investigations that employ more robust research designs and data collection methods to enhance the understanding of social participation among persons with visual impairment.

## 5. Conclusion

The factors affecting the social participation of people with visual impairment based on the PSED data were analyzed in this study. The variables affecting the social participation of persons with visual impairment included the stability of employment, job satisfaction, and monthly income. Therefore, the aim of this study is to serve as a foundational dataset for future approaches and studies within the field of occupational therapy, with the goal of enhancing social participation among people with visual impairment.

## Figures and Tables

**Table 1:** General characteristics of study subjects (*n* = 151).

		*n*	%
Sex	Male	112	74.2
	Female	39	25.8

Age	15-29	1	00.7
	30-39	23	15.2
	40-49	43	28.5
	50-59	45	29.5
	60-68	39	25.8

The level of education	Less than middle school graduation	29	19.2
	High school graduation	64	42.4
	More than university graduation	58	38.4

Disability severity	Mild	130	86.1
	Severe	21	13.9

**Table 2:** Results of correlation analysis among variables.

	Social participation	Daily life satisfaction	Job satisfaction	Gender	Age	Education level
Daily life satisfaction	.297^∗∗∗^					
Job satisfaction	.310^∗∗^	.463^∗∗∗^				
Gender	-.060	-.034	.041			
Age	-.157	-.218^∗∗^	-.141	-.019		
Education level	.129	.108	.117	-.072	-.422^∗∗∗^	
Disability severity	.075	.029	-.069	-.069	.085	-.025

^∗∗^ *p* < .01, ^∗∗∗^*p* < .001.

**Table 3:** Causal relationship between subfactors of daily life satisfaction and social participation.

	Unstandardized coefficients		Standardized coefficients	*t*	Tolerance	VIF
	*B*	S.E	*B*			
Constant	1.872	.199		9.425^∗∗∗^		
Monthly income	.195	.059	.260	3.292^∗∗^	1.00	1.00
*R* ^2^	.362					
*F*(*p*)	10.840^∗∗∗^					

^∗∗^ *p* < .01, ^∗∗∗^*p* < .001.

**Table 4:** Causal relationship between subfactors of job satisfaction and social participation.

	Unstandardized coefficients		Standardized coefficients	*t*	Tolerance	VIF
	*B*	S.E	*B*			
Constant	1.619	.271		5.977^∗∗∗^		
Stability of employment	.252	.075	.309	3.371^∗∗^	1.00	1.00
*R* ^2^	.387					
*F*(*p*)	11.367^∗∗∗^					

^∗∗^ *p* < .01, ^∗∗∗^*p* < .001.

**Table 5:** Causal relationship among variables affecting social participation.

	Unstandardized coefficients		Standardized coefficients	*t*	Tolerance	VIF
	*B*	S.E	*B*			
Constant	1.177	.397		2.963^∗∗∗^		
Job satisfaction	.159	.011	.310	3.394^∗∗^	1.00	1.00
*R* ^2^	.388					
*F*(*p*)	11.519^∗∗∗^					

^∗∗^ *p* < .01, ^∗∗∗^*p* < .001.

## Data Availability

The data used to support the findings of this study are available from the corresponding author upon request.
